# Application Value of Emergency Bedside Echocardiography in Early Warning of Acute and Severe Shock and Clinical Classification

**DOI:** 10.1155/2022/1634866

**Published:** 2022-07-19

**Authors:** Juan Ye, Yan Lin, Shaolin Chen

**Affiliations:** ^1^Ultrasound Imaging Department, The First People's Hospital of Jiangxia, Wuhan City, Hubei Province 430200, China; ^2^Department of Emergency, Shenzhen People's Hospital, The Second Clinical Medical College, Jinan University; The First Affiliated Hospital, Southern University of Science and Technology, Shenzhen, 518020 Guangdong, China

## Abstract

**Objective:**

A case-control study was conducted to explore the application value of emergency bedside echocardiography in early warning of acute and severe shock and clinical classification.

**Methods:**

A total of 135 critically ill patients admitted to ICU from August 2019 to November 2020 were divided into shock group (*n* = 53) and nonshock group (*n* = 82) according to the occurrence of shock. The internal diameter index of inferior vena cava was measured and recorded by bedside ultrasound in patients with shock before and after treatment and in patients without shock. Shock index and inferior vena cava diameter deformation index (SCI) were calculated according to the results. The diagnostic time and curative effect of different ultrasonic examination methods for the types of shock were compared and analyzed.

**Results:**

At admission, the maximum and minimum ventilation of inferior vena cava in patients without shock were higher than those in the shock group, and the internal diameter deformation index of inferior vena cava in the shock group was higher than that in the shock group (*P* < 0.05). In the shock group, IVCmax and IVCmin before and after treatment were higher than those before resuscitation, while SCI was lower than that before resuscitation. The results of ROC curve analysis showed that SCI and IVCmin were significantly better than IVCmax and IVCmin in predicting shock area and slightly better than IVCmin. There was significant difference in diagnosis time between the two groups (*P* < 0.05). The specificity, positive predictive value, and negative predictive value of emergency ultrasound diagnosis were lower than those of clinical diagnosis (*P* < 0.05). The sensitivity, specificity, positive predictive value, and negative predictive value of emergency ultrasound diagnosis were lower than those of clinical diagnosis (*P* < 0.05). The sensitivity and positive predictive value of the emergency ultrasound group were higher than those of the routine ultrasound group (*P* < 0.05). The diagnosis rate of shock type AUC in the emergency ultrasound group was 0.854, and the diagnostic value was high.

**Conclusion:**

IVCmax, IVCmin, and SCI obtained by bedside ultrasound have certain clinical significance for the diagnosis and treatment of shock. Emergency bedside ultrasound examination and measurement of shock patients are helpful to quickly evaluate and identify the types of early shock.

## 1. Introduction

Shock is one of the most obvious acute and critical diseases in the emergency department, which refers to a significant decrease in systemic effective circulatory blood volume and a sharp decrease in tissue and organ perfusion due to various reasons (such as massive hemorrhage, burn infection, and heart pump failure) [1]. The clinical pathophysiological processes leading to histiocytic hypoxia and organ dysfunction may induce stroke. Despite the continuous innovation of medical technology, the early diagnosis and correct intervention of shock are still major challenges for emergency doctors.

The existing examination methods mainly rely on monitoring blood pressure, heart rate, cardiac index, CVP, pulmonary artery wedge pressure (PAWP), and other hemodynamic tests to diagnose shock [2]. For example, the important marker of decompensation stage of shock is the decrease of CVP. Shock treatment with CVP monitoring can effectively reduce the possibility and mortality of arrhythmias during resuscitation [3]. It is an important detection method commonly adopted in clinical treatment. However, because the CVP monitoring needs to give patients deep venipuncture catheterization, because it is invasive and difficult to operate, it often cannot be completed in the first time in the event of traumatic hemorrhagic shock. It is difficult for doctors to objectively and accurately evaluate the hemodynamics of patients in time.

At present, bedside ultrasound diagnostic instruments are more often adopted for emergency ultrasound examination [4]. Although the imaging function of bedside ultrasound is slightly weaker, and the development of fine structure is not as good as large ultrasound, compared with other examination methods, bedside ultrasound has obvious advantages in hemodynamic evaluation of patients and has the advantages of portability, rapidness, and ease of operation. Bedside ultrasound can provide items such as ultrasound-guided diagnostic puncture, detection of pleural and peritoneal effusion, echocardiography, diameter measurement of aorta, and superior and inferior vena cava in the diagnosis and treatment of acute and severe shock [5]. There is no valve in the superior and inferior vena cava, which has excellent compliance, and its diameter is easy to change with the change of effective circulatory blood volume. Ultrasonic evaluation will reflect the hemodynamic abnormality during shock to some extent [6]. Compared with the superior vena cava, the inferior vena cava has a longer diameter and simpler surrounding anatomical structure, and the inferior vena cava collects blood from the abdominal cavity and lower limbs, and its blood flow is more compared to the superior vena cava, which is easier to reflect the change of circulating blood volume [7]. However, at present, the more reliable ultrasonic evaluation of the cause of shock is mainly to evaluate the cardiopulmonary condition, and the ultrasonic evaluation of large vessels is not adopted as an independent means to diagnose the state of shock, and there is no quantitative standard for the evaluation of the examination results. And there is no sufficient and strong evidence to prove that it can be adopted as a reliable and independent diagnostic method to judge the state of acute and severe shock and to monitor the process of fluid resuscitation [8]. Based on this, 135 critically ill patients admitted to ICU in our hospital from March 2019 to August 2020 were studied, which are reported as follows.

## 2. Patients and Methods

### 2.1. General Information

A total of 135 critically ill patients admitted to ICU from August 2019 to November 2020 were assigned into shock group (*n* = 53) and nonshock group (*n* = 82) according to the occurrence of shock. The age of the shock group was 18-88 years old, and that of the nonshock group was 19-89 years old. There exhibited no statistical difference in general data, as indicated in Table 1. This study was permitted by the Medical Ethics Association of our hospital.

Selection criteria are as follows: (1) patients with noncardiac surgery admitted to ICU and patients with stay in ICU≧24 hours regardless of gender, (2) complete clinical data, and (3) informed consent was signed by all patients or their legal representatives.

Exclusion criteria are as follows: (1) eliminate severe visual and auditory impairment and be unable to communicate with visitors; (2) congenital heart disease, valvular heart disease, right heart failure, pericardial tamponade, and pulmonary hypertension; (3) refuse to participate; (4) those who are not expected to survive for more than 24 hours; (5) irritability and hyperactivity cannot cooperate with or cannot take the supine position, and the abdominal injury is in the contact area of ultrasonic examination; (6) those with incomplete clinical data.

### 2.2. Treatment Methods

#### 2.2.1. Data Acquisition

(1) General data: the diagnosis, age, sex, height, weight, blood pressure, and heart rate at different times were recorded; (2) IVC pipe diameter: use Mindray M7 super portable ultrasound instrument, P4-2S probe and frequency 2~5 MHz equipped in emergency department of our hospital. Make the patient take supine position, choose M mode of ultrasonic instrument, put the probe in the best position of IVC imaging under xiphoid process, carry out ultrasonic examination from horizontal position, freeze the ultrasonic image of IVC cross section when the maximum deformation occurs at the end of inspiration, and measure that the IVC cross section is an approximate ellipse with a certain inclination angle between the long axis and the coronal plane of the body, and take the long axis and short axis of the ellipse as the maximum and minimum diameter of the IVC to record its length.

The patients in the shock group recorded the state of hemorrhagic shock and corrected shock by fluid resuscitation, operation, or other treatment, the vital signs were stable, and the IVC diameter data were collected only once when the trauma patients without shock were admitted to the hospital. During ultrasound examination, IVCmax and IVCmin were measured 3 times, respectively, and the mean value was taken and recorded. The whole process is completed by the same operator, and the measuring time is controlled within 10 minutes. (3) All patients in the shock group had deep vein catheterization. CVP data were measured before fluid resuscitation treatment and in the meantime as ultrasound data were collected. When the patient's condition and vital signs are stable after rescue and surgical treatment, the CVP value is measured again. Patients who do not meet the criteria and diagnosis of hemorrhagic shock are often not given invasive deep venipuncture catheterization and do not measure CVP. (4) Count the diagnosis time of patients (min, from the emergency department doctor to the diagnosis time).

### 2.3. Statistical Analysis

The data are analyzed and processed by the SPSS25.0 and MedCalc19.7.2 statistical software. The measurement data in accordance with normal distribution are presented as (*x* ± *s*), and the adoption rate and constituent ratio of counting data are presented. As a case-control group of critically ill patients, chi-square test was adopted to compare the count data between sample groups, and independent sample *t*-test was employed to measure data. Paired sample *t*-test was adopted to compare the data of patients with shock, and the correlation test of each data was verified by Pearson correlation coefficient. ROC curve was adopted to analyze the effect of IVC diameter-related data in predicting shock state and the diagnostic efficacy of different ultrasound diagnostic criteria. The DeLong test of the Med Calc software was adopted to analyze the difference of ROC curve. *P* < 0.05 was defined as statistically significant.

## 3. Results

### 3.1. Comparative Analysis of General Data of Patients

The general data were analyzed. A total of 135 patients with severe ICU were included. According to the occurrence of shock, the incidence of shock was 39.26% (53/135). There exhibited no significant difference in sex, age, height, weight, and BMI between two groups (*P* > 0.05). There were significant differences in heart rate, blood pressure, and shock index at admission between two groups (*P* < 0.05). All the results are indicated in Table 1.

### 3.2. Comparison of Corrected IVC Indexes between Nonshock Group and Shock Group

The corrected IVC indexes of the nonshock group and the shock group were compared. IVCmax, IVCmin, and SCI were compared between the nonshock group and the shock group as baseline. There exhibited no significant difference between two groups (*P* > 0.05). All the results are indicated in Table 2.

### 3.3. Comparison of IVC Indexes at Admission

The IVC indexes at admission were compared. IVCmax and IVCmin in patients without traumatic shock were higher compared to the shock group, while the SCI was lower compared to the shock group. There exhibited significant difference before and after (*P* < 0.05). All the results are indicated in Table 3.

### 3.4. Comparison of IVC Indexes in Shock Group before and after Treatment

We compared the IVC before and after treatment in the shock group. The IVCmax and IVCmin of the shock group before and after treatment were higher than those before resuscitation, and SCI was lower than that before resuscitation. There exhibited significant difference before and after (*P* < 0.05). All the results are indicated in Table 4.

### 3.5. Analysis of ROC Curve between Shock Group and Nonshock Group

Using ROC curve for statistical analysis, the results show that SCI and IVCmin are remarkably better than IVCmax and SCI and slightly better than IVCmin in predicting shock in terms of AUC area. The cutoff value was 2.05 cm for IVCmax, 1.29 cm for IVCmin, and 1.43 for SCI. By DeLong test, there was no significant difference in predictive performance between SCI and IVCmin (*P* > 0.05). The results are indicated in Table 5 and Figure 1.

### 3.6. Comparison of Diagnostic Time between Conventional Ultrasound and Emergency Ultrasound

In terms of emergency ultrasound, the diagnosis time of conventional ultrasound was the longest (14 min), with an average of 12.34 ± 1.16 min. The diagnosis time of emergency ultrasound was the longest (10 min), averaging 8.34 ± 1.06 min. There exhibited significant difference in diagnosis time (*P* < 0.05).

### 3.7. Effectiveness Analysis of Two Diagnostic Criteria

The sensitivity, specificity, positive predictive value, and negative predictive value of the emergency ultrasound group were 100.00%, 78.92%, 21.13%, and 0, respectively. The diagnostic specificity, positive predictive value, and negative predictive value were lower compared to clinical diagnosis (all *P* < 0.05). The sensitivity, specificity, positive predictive value, and negative predictive value of the conventional ultrasound group were 91.46%, 96.09%, 3.91%, and 8.54%, respectively. The diagnostic sensitivity, specificity, positive predictive value, and negative predictive value were lower compared to clinical diagnosis (*P* < 0.05). With regard to different ultrasound methods, the sensitivity and positive predictive value of the emergency ultrasound group were higher compared to the conventional ultrasound group (*P* < 0.05). Further comparing the diagnostic efficacy of different ultrasound methods, the ROC curve indicated that the AUC of the emergency ultrasound group in diagnosing the type of shock was 0.854, which was of higher diagnostic value, as indicated in Table 6 and Figure 2 for details.

## 4. Discussion

Most of the patients with acute and severe shock are complicated and serious, and it is difficult to tolerate the cooperation of invasive operation which takes a long time, and most of the patients with multiple injuries have poor skin condition at the puncture site, which belongs to the contraindication of puncture operation [8–10]. CVP data are also easily affected by cardiopulmonary diseases, vascular tension, changes of blood biochemical indexes, and increase or decrease of thoracic and abdominal pressure. CVP and shock index are adopted in isolation to guide emergency rescue of patients with traumatic shock. It is not recommended in recent national and international guidelines for trauma diagnosis and treatment [11–14]. While bedside ultrasound examination, the use time of collecting each index of inferior vena cava diameter is much shorter than other invasive hemodynamic detection methods, and there is no risk of secondary injury to the tissue [15].

Bedside ultrasound can measure and calculate the IVCmax, IVCmin, and SCI of patients, judge the blood volume of patients, so as to early judge the state of shock, and guide emergency fluid resuscitation treatment [16]. As the vein with the largest blood flow in the human body, the inferior vena cava has a good correlation with the CVP, so it can be adopted to evaluate the blood volume of the body during shock [17]. The trunk of inferior vena cava is longer compared to superior vena cava and can be easily measured by ultrasound [18]. When the human body lies flat, the cross section of the inferior vena cava is approximately oval, which can be deformed with the movement of breathing. During the occurrence of shock, with the decrease of effective circulating blood volume, the filling pressure in the inferior vena cava decreased, the tube diameter became smaller, and the cross section decreased. Related studies have indicated that the cross-sectional shape of the inferior vena cava seen in computed tomography is related to the effective circulatory blood volume of the patient [19]. However, the CT image is an instantaneous examination result, which cannot be used to judge which respiratory phase the inferior vena cava is in. Moreover, the cost of CT examination is high, the radioactivity is strong, and the examination equipment is limited by the environment, so it cannot dynamically monitor the changes of blood volume in patients with shock. In an abdominal ultrasonography, it is easy to obtain the image of inferior vena cava, and the abdominal segment under xiphoid process and right midaxillary line can be adopted as ultrasonic probe. In the meantime, ultrasound can dynamically observe the shape changes of the cross section of the inferior vena cava, freeze the examination images in different breathing phases, and measure the diameter of the cut inferior vena cava immediately. The inferior vena cava diameter deformation index (SCI) is a ratio, which can reflect the degree of deformation of the inferior vena cava with respiratory movement, and to some extent, it can eliminate the influence caused by the great difference in body shape, such as body height and weight, and can be adopted as a key index for monitoring the changes of circulating blood volume during fluid therapy [20].

By monitoring the diameter of inferior vena cava by bedside ultrasound, SCI can be calculated and evaluated in real time, noninvasive, convenient, and easy to repeat, so as to understand the blood volume of patients, so as to adjust the speed and scheme of fluid replacement in time, and play an important role in the clinical treatment of hemorrhagic shock in traumatic patients [21–24]. The first time is to understand the physical injury of patients, further shorten the time of rescue and treatment, enhance the survival of patients, promote the prognosis of trauma patients, and optimize the level of medical treatment.

In this study, it was found that the IVC indexes at admission were higher compared to the shock group, while the SCI was lower compared to the shock group (*P* < 0.05). Comparison of IVC before and after treatment in the shock group indicated that IVCmax and IVCmin in the shock group before and after treatment were higher than those before resuscitation, while SCI was lower than that before resuscitation (*P* < 0.05). In terms of AUC area, SCI and IVCmin were remarkably better than IVCmax and SCI and slightly better than IVCmin, in predicting the occurrence of shock. The cutoff value was obtained. IVCmax was 2.05 cm, IVCmin was 1.29 cm, and SCI was 1.43. The DeLong test results show that the prediction efficiency of SCI is equivalent to that of IVCmin. In addition, compared with emergency ultrasound, the diagnosis time of conventional ultrasound was the longest (14 min) and that of emergency ultrasound was the longest (10 min) (*P* < 0.05). The sensitivity and positive predictive value of the emergency ultrasound group were higher compared to the routine ultrasound group (all *P* < 0.05). Thus, it can be noticed that the inferior vena cava diameter data obtained by bedside color Doppler ultrasound can diagnose and predict the occurrence of shock more accurately than shock index, blood pressure, heart rate, and other noninvasive detection methods.

When studying the effect of emergency doctors using severe ultrasound to identify early shock types, some scholars Chandra et al. confirmed that emergency doctors can identify early shock types more quickly and accurately and improve the quality of medical treatment [25]. According to the study of Choi et al. in the clinical practice of emergency ultrasound in the study of unexplained shock, through the analysis of several cases of diagnosis and treatment of patients with unexplained shock, it is proved that emergency doctors can quickly identify the shock types of acute and critically ill patients with severe shock, then clear to the etiological diagnosis and timely and correct rescue, and improve the poor prognosis [26]. In the meantime, Shi and other scholars also confirmed that cardiopulmonary ultrasound can not only make a definite diagnosis but also rule out the causes of shock, such as pericardial tamponade, pulmonary embolism, pneumothorax, and heart failure. More importantly, emergency doctors can not only quickly identify the types of early shock by severe ultrasound but also evaluate the hemodynamic response by observing the imaging changes of heart and lung by severe ultrasound to achieve visual and accurate rehydration [27–29]. The results of this study show that the AUC of the diagnostic ultrasound group for the diagnosis of shock type is 0.854, which is of high diagnostic value, which is basically consistent with the conclusions of previous studies. The same idea can be found in the study put forward by Wang et al. [30]. They have applied new methods in the study, and the conclusions drawn can also give some support to this study.

To sum up, the lumen diameter of IVC is more affected by its internal blood flow. During the period of early shock and body compensation, the diameter of inferior vena cava can more sensitively and specifically reflect the abnormality of blood circulation in patients. Emergency doctors use severe ultrasound to examine patients in the early stage of shock, which can quickly and accurately identify the type of shock, timely and correct treatment, safe and reliable, economical, and portable and can be widely adopted in clinic.

## Figures and Tables

**Figure 1:** ROC curve of IVC parameters.

**Figure 2:** ROC of emergency ultrasound diagnosis of shock types.

**Table 1:** Comparison of general data of critically ill inpatients.

General data	Shock group (*n* = 53)	Nonshock group (*n* = 82)	*t*/*χ*^2^	*P*
Gender (male/female)	26/27	44/38	0.273	>0.05
Age (years)	45.62 ± 12.12	46.46 ± 13.25	0.372	>0.05
Height (cm)	167.65 ± 9.65	166.89 ± 9.52	0.360	>0.05
Body weight (kg)	70.38 ± 20.27	65.68 ± 9.77	1.803	>0.05
BMI (kg/m^2^)	24.88 ± 5.35	23.74 ± 2.56	1.660	>0.05
Heart rate (beats/min)	116.27 ± 13.28	90.18 ± 17.15	9.398	<0.05
Systolic blood pressure (mmHg)	92.18 ± 10.69	122.89 ± 19.23	10.606	<0.05
Diastolic pressure (mmHg)	56.85 ± 11.04	76.59 ± 14.11	8.618	<0.05
Shock index	1.26 ± 0.24	0.79 ± 0.16	13.660	<0.05

Note: There exhibited no significant difference in sex, age, height, weight, and BMI (*P* > 0.05). There were significant differences in heart rate, blood pressure, and shock index at admission (*P* < 0.05).

**Table 2:** Comparison of IVC indexes without shock (*x̅*±*S*).

Grouping	*N*	IVCmax (cm)	IVCmin (cm)	SCI
Shock group (correction)	53	2.03 ± 0.14	1.55 ± 0.22	1.36 ± 0.25
Nonshock group	82	2.01 ± 0.11	1.53 ± 0.14	1.34 ± 0.07
*t*		0.926	0.646	0.685
*P*		>0.05	>0.05	>0.05

Note: There exhibited no significant difference between two groups (*P* > 0.05).

**Table 3:** Comparison of IVC indexes at admission.

Grouping	*N*	IVCmax (cm)	IVCmin (cm)	SCI
Shock group (correction)	53	1.91 ± 0.15	0.97 ± 0.41	2.48 ± 1.24
Nonshock group	82	2.03 ± 0.11	1.51 ± 0.13	1.33 ± 0.06
*t*		5.355	11.113	8.400
*P*		<0.05	<0.05	<0.05

Note: There exhibited significant difference before and after (*P* < 0.05).

**Table 4:** Comparison of IVC indexes in the shock group before and after treatment.

Grouping	*N*	IVCmax (cm)	IVCmin (cm)	SCI
Before treatment	53	1.89 ± 0.13	0.97 ± 0.41	2.45 ± 1.23
After treatment	53	2.03 ± 0.12	1.56 ± 0.23	1.31 ± 0.22
*t*		5.761	9.137	6.642
*P*		<0.05	<0.05	<0.05

Note: There exhibited significant difference before and after (*P* < 0.05).

**Table 5:** ROC analysis of IVCmax, IVCmin, and SCI in predicting traumatic hemorrhagic shock.

Index	Sensitivity degree (%)	Specificity (%)	AUC	95% CI
IVCmax	48.31	90.02	0.711	0.558~0.863
IVCmin	72.03	98.23	0.891	0.799~0.982
SCI	80.05	94.45	0.931	0.847~0.999

Note: The cutoff value was 2.05 cm for IVCmax, 1.29 cm for IVCmin, and 1.43 for SCI. By DeLong test, there was no significant difference in predictive performance between SCI and IVCmin (*P* > 0.05).

**Table 6:** Comparison of emergency bedside ultrasound and clinical diagnosis.

Results of auxiliary examination or clinical diagnosis	*N*	Emergency bedside ultrasound		Conventional ultrasound	
		Positive	Negative	Positive	Negative
Positive	53	53	0	48	5
Negative	82	17	65	22	60
Total	135	70	65	70	65

Note: The diagnostic sensitivity, specificity, positive predictive value, and negative predictive value were lower compared to clinical diagnosis (*P* < 0.05). With regard to different ultrasound methods, the sensitivity and positive predictive value of the emergency ultrasound group were higher compared to the conventional ultrasound group (*P* < 0.05).

## Data Availability

The datasets used and analyzed during the current study are available from the corresponding author upon reasonable request.
